The article "Rutin and Quercetin Counter Doxorubicin-Induced Liver Toxicity in Wistar Rats via Their Modulatory Effects on Inflammation, Oxidative Stress, Apoptosis, and Nrf2" was published in 2022. Journal: Oxid Med Cell Longev.

# Rutin and Quercetin Counter Doxorubicin-Induced Liver Toxicity in Wistar Rats *via* Their Modulatory Effects on Inflammation, Oxidative Stress, Apoptosis, and Nrf2

**DOI:** 10.1155/2022/2710607

**Published:** 2022-07-27

**Authors:** Osama M. Ahmed, Mohammed H. Elkomy, Hanaa I. Fahim, Mohamed B. Ashour, Ibrahim A. Naguib, Badrah S. Alghamdi, Heba Uallah R. Mahmoud, Noha A. Ahmed

**Affiliations:** ^1^Physiology Division, Zoology Department, Faculty of Science, Beni-Suef University, P.O. Box 62521, Beni-Suef, Egypt; ^2^Department of Pharmaceutics, College of Pharmacy, Jouf University, Sakaka 72341, Saudi Arabia; ^3^Department of Pharmaceutical Chemistry, College of Pharmacy, Taif University, P.O. Box 11099 Taif 21944, Saudi Arabia; ^4^Department of Physiology, Neuroscience Unit, Faculty of Medicine, King Abdulaziz University, Jeddah 22252, Saudi Arabia; ^5^Pre-Clinical Research Unit, King Fahd Medical Research Center, King Abdulaziz University, Jeddah, Saudi Arabia

## Abstract

The presented study was performed to verify whether rutin and/or quercetin can inhibit liver injury induced by doxorubicin (DXR) in male Wistar rats. In this study, male Wistar rats were treated via the oral route with rutin and quercetin (50 mg/kg) either alone or in combination every other day for five weeks concomitant with receiving intraperitoneal DXR (2 mg/kg) two times a week for five successive weeks. Quercetin, rutin, and their combination significantly improved the deteriorated serum AST, ALT, and ALP activities and total bilirubin level, as well as albumin, AFP, and CA 19.9 levels in DXR-injected rats. Treatments of the DXR-injected group with quercetin and rutin prevented the elevation in liver lipid peroxidation and the reduction in superoxide dismutase, glutathione-S-transferase and glutathione peroxidase activities, and glutathione content. Treatments with quercetin and rutin significantly repressed the elevated expression of liver p53 and TNF-*α* and enhanced Nrf2 expression. Furthermore, the treatments significantly reduced DXR-induced liver histological changes. In conclusion, rutin and quercetin either alone or in combination may have potential preventive effects against DXR-induced hepatotoxicity through inhibiting oxidative stress, inflammation, and apoptosis as well as modulating the Nrf2 expression.

## 1. Introduction

Doxorubicin (DXR) is an anthracycline antibiotic with broad spectrum activity and is considered one of the most effective chemotherapeutics against cancer [1]. It is used alone or in combination to treat a variety of hematological and solid malignancies, including breast cancer [2]. Despite its therapeutic efficacy, DXR is accompanied by notable liver toxicity and other organ toxicities [3–9], which may limit the scope of its clinical applications in the treatment of cancer. Additionally, DXR counters cell proliferation, activates oxidative stress, attenuates antioxidant defense system, suppresses topoisomerase type II, and eventually results in cells' death due to necrosis or apoptosis [10–12]. Although inflammation, apoptosis, deoxyribonucleic acid (DNA) damage, calcium metabolism impairment, and excessive free radical production may have a direct effect in the degeneration of organ function to varying degrees, the specific mechanism of DXR-mediated multiple organ toxicity has not yet been fully investigated [13]. DXR accumulates in the mitochondria, causing structural and functional alterations. Nevertheless, elevation of reactive oxygen species (ROS) and reactive nitrogen species (RNS) to substantial levels within the cell, which finally leads to cell damage and programmed cell death (PCD), is regarded as one of the main reasons of DXR-induced adverse effects in humans and animals [14, 15]. When the amount of ROS produced within a cell surpasses its defense requirement, the cell is declared in “oxidative stress” state. Induction of protein oxidation and lipid peroxidation (LPO), inhibition of antioxidant enzymes, nucleic acid injury, PCD pathway stimulation, and eventual cell death or damage are among the hazards created by increased liberation of ROS evoked by environmental conditions [16, 17]. Connection between oxidative stress and DXR-induced toxicity has been established in various body organs [7, 18]. As a result, using antioxidants [7, 8] such as natural flavonoids together with DXR may help decrease or prevent DXR-induced adverse effects.

Plant constituents with aromatic ring in their core structure and one or more hydroxyl groups are known as flavonoids beside other phenolic substances. Of these constituents, >8000 phenolic compounds have been identified [19, 20]; of which, 50% are flavonoids (glycosides, aglycones, and methylation derivatives) [21]. These phytochemical compounds can be found in foods and herbal medications. The flavonoids and various other reported phenolic components were found to exhibit excellent antioxidative, cardioprotective, anticancer, antibacterial, antidiabetic, antihypertensive, anti-inflammatory, and immune response boosting effects and provide skin protection from hazardous ultraviolet radiation (UV) radiation, making them outstanding drugs for pharmaceutical and medical use [22–24]. The flavonoid quercetin has a glycoside known as rutin (quercetin rutinoside). It works as an antioxidant in humans by connecting to the ferrous iron **(**Fe^+2^), thus preventing generation of highly reactive free radicals which might harm cells [4]. Rutin has also been shown to produce anti-inflammatory effect *in vitro* and in animal models [25]. Moreover, renocardioprotective, antidiabetic, and anticancer properties have been reported for rutin [8, 24, 26]. Quercetin, which is known as a natural plant-derived aglycone of rutin, is frequently used as a dietary supplement and was recently shown to be effective in the treatment of several diseases. Cardiovascular protective, renocardioprotective, anticancer, antiulcer, antiallergy, anti-inflammatory, antiviral, antidiabetic, antihypertensive, gastroprotective, immunomodulatory, and anti-infective qualities are only a few of quercetin beneficial effects [8, 24, 27, 28]. In our previous publication, rutin and quercetin, *via* suppressing oxidative stress and boosting antioxidant defense system, were labeled as chemopreventive agents against nephrocardiotoxicity induced by doxorubicin [8]. Most of other publications investigated the effects of rutin and quercetin on DXR-induced cardiotoxicity [29–33], but rare published studies assessed their effects on DXR-induced hepatotoxicity [34, 35]. However, the mechanisms of actions were not entirely delineated by these studies. Furthermore, no published studies have revealed the combinatory effects of rutin and quercetin on DXR-induced hepatotoxicity.

Therefore, the presented study was designed to determine whether rutin and quercetin, as well as their combination, could help to prevent DXR-induced liver damage and toxicity in a male Wistar rat animal model.

## 2. Materials and Methods

### 2.1. Experimental Animals

In the presented study, 50 male Wistar rats weighing approximately 120-145 g (about 10 weeks old) were selected as experimental animals. They were obtained from the “National Research Center's Animal House in Giza, Egypt.” The experimental animals were adapted to laboratory set conditions for 10 days prior to experiments. The rats were accommodated in polyethylene cages withheld under room temperature set to 25 ± 1°C and relative humidity set to 20%-30% with cyclic daylight (12 h/day). The animals were granted free full access to drinking water and were supplemented balanced commercial pelleted diet. The Ethics Committee of the Care and Use of Experimental Animals, Faculty of Science, Beni-Suef University, Egypt, has approved the experimental study (ethical approval number: BSU/FS/2015/22). All attempts have been made to reduce pain and discomfort.

### 2.2. Chemicals and Drugs

Pharmacia Italia (Milan, Italy) provided the DXR in the form of Adriamycin hydrochloride. Sigma Chemical Company (St. Louis, MO, USA) provided the rutin and quercetin. All of the other chemicals were ultrapure and available at market.

### 2.3. Doses and Treatment

DXR was administered intraperitoneally to the animals. The dose of DXR was adjusted to 2 mg/1 mL sterile isotonic saline/kg bw (kilogram body weight) [7, 8] and given twice a week for 5 weeks. The doses of quercetin and rutin were modified to 50 mg/kg bw [36, 37] and given orally every other day for 5 successive weeks *via* oral gavage. Drug solutions in carboxymethyl cellulose (CMC) were prepared by solvating rutin or quercetin (50 mg) in 1% CMC (5 mL).

### 2.4. Animal Grouping

In this experiment, the rats were categorized into five separate groups (10 rats for each) as indicated in Scheme 1:

Group 1 (normal group): for 5 successive weeks, this group was intraperitoneally injected with sterile isotonic saline (1 mL/kg) every other day. During the same period on every other day, the group was also given 5 mL/kg of 1% CMC by oral administration

Group 2 (DXR-injected control group): for 2 days per week for 5 successive weeks, DXR (2 mg/kg) was given to this group intraperitoneally [7, 8]. Moreover, for 5 successive weeks on every other day, this group was also given 5 mL/kg of 1% CMC by oral administration

Group 3 (DXR-injected group supplemented with rutin): similar to the DXR-injected control group, this group was given DXR intraperitoneally. Moreover, for 5 successive weeks, this group was given rutin (50 mg/kg bw) orally every other day [36]

Group 4 (DXR-injected group supplemented with quercetin): similar to the DXR-injected control group, this group was given DXR intraperitoneally. Moreover, for 5 successive weeks, this group was given quercetin (50 mg/kg bw) orally every other day [37]

Group 5 (DXR-injected group supplemented with rutin and quercetin): similar to the DXR-injected control group, this group was given DXR intraperitoneally. Moreover, for 5 successive weeks, this group was orally coadministered with rutin (50 mg/kg bw) and quercetin (50 mg/kg bw) every other day

### 2.5. Tissue and Blood Sampling

Blood samples were taken from each rat's jugular vein at the end of the experiment after induction of anesthesia *via* diethyl ether inhalation. The samples were then stored in centrifuge tubes and let to coagulate for 45 minutes (min) at ambient temperature before being centrifuged for 15 min at 3000 rpm. For every animal, the collected sera (clear, nonhemolyzed supernatant) were split into 4 sections and stored at -30°C for subsequent biochemical analysis. The animals were then sacrificed and dissected for isolation of the liver. The isolated levers were homogenized separately in 10% *w*/*v* phosphate-buffered saline solution (pH 7.2) using a Telfon homogenizer (Glas-Col, Terre Haute, USA). After centrifugation of the collected homogenates at 3000 rpm (round per min), the obtained supernatants were then extracted and fractionated into 3 sections, which were maintained in a deep freezer (at -30°C) till utilized for measurement of antioxidant defense markers and oxidative stress.

### 2.6. Biochemical Studies

The method of Murray was adopted to assess serum alanine transaminase (ALT) and aspartate transaminase (AST) [38] utilizing the reagent kits acquired from Spinreact (Spinreact, S.A./S.A.U. Ctra.Santa Coloma, 7 E-17176 Sant Esteve De Bas (Gi) Spain). Serum alkaline phosphatase (ALP) was measured according to the method of Schumann et al. [39] utilizing the reagent kits acquired from Spectrum Diagnostics (Al-Obour City, Cairo, Egypt). The total bilirubin in the serum was measured through a colorimetric process using Spectrum Diagnostics kits according to Balistreri and Shaw [40]. According to Gendler [41], serum albumin was tested using a colorimetric method utilizing the kits acquired from Diamond Diagnostics (24 El Mon-tazah St., Heliopolis, Cairo, Egypt). The serum tumor markers, alpha fetoprotein (AFP), and carbohydrate antigen 19.9 (CA19.9), were quantitatively measured employing the enzyme immunosorbent assay (ELISA) and using kits acquired, respectively, from R&D Systems, Inc. (614 McKinley Place NE, Minneapolis, MN 55413, USA) and RayBiotech, Inc. (3607 Parkway Lane, Suite 100 Norcross, GA 30092) in accordance with the instructions supplied with each kit.

The levels of malondialdehyde (MDA) as an indicator of LPO [42], glutathione peroxidase (GPx) [43], glutathione (GSH) [44], superoxide dismutase (SOD) [45], and gluathione-S-transferase (GST) [46] of the liver were assessed according to published methods.

### 2.7. Immunohistochemical Investigation

For immunohistochemical detection of apoptotic protein (p53), tumor necrosis factor-*α* (TNF-*α*), and nuclear factor erythroid 2–related factor 2 (Nrf2), pieces of liver (3 mm^3^) were fixed in 10% NBF (neutral-buffered formalin). The fixed liver samples were processed, blocked, and sectioned into 5 *μ*m thick sections that were then mounted onto positive-charged slides (Fisher Scientific, Pittsburgh, PA, USA) in the Department of Pathology, National Cancer Institute (NCI), Cairo University, Egypt. The reactivity of p53 and Nrf2 was investigated using the methods of previous publications [47–52]. Dilution of the primary antibody was 1 : 100 in phosphate buffer saline (PBS) and dilutions of the secondary biotinylated antibodies of p53 and Nrf2 were, respectively, 1 : 100 and 1 : 200 in PBS. ImageJ, a free software program, was used to examine and analyze the labeling (1.51 d) [53]. The integrated intensities (in pixels) of the positive reaction of p53 and Nrf2 were measured using ImageJ software.

### 2.8. Histopathological Studies

Pieces of the liver (3 mm^3^) from each tested animal were transported to the “Pathology Department, NCI, Cairo University, Egypt” after preserving in 10% NBF. The samples were processed and stained with hematoxylin and eosin (H&E) based on the technique revealed by Banchroft et al. [54]. The stained liver sections were then inspected by a histopathologist to detect histopathological lesions. Lesions were scored and graded 0 (absence of lesion), I (mild), II (moderate), or III (severe).

### 2.9. Statistical Analysis

The obtained data were represented as mean ± standard error of mean (*M* ± SEM). One-way analysis of variance (ANOVA) was employed for data analysis using PC-STAT statistical program [55]. For each variable, pairwise comparisons of different groups were achieved by employing the least significant difference (LSD) post hoc test at *P* < 0.05 and *P* < 0.01.

## 3. Results

### 3.1. Effect on Liver Function Relevant Serum Parameters

The data representing the effect on serum ALT, AST, and ALP activities as well as on the albumin levels and total bilirubin by quercetin and/or rutin is shown in Table 1. The intraperitoneal administration of DXR to rats resulted in a significant elevation (*P* < 0.01) in the activities of serum ALT (75.65%), AST (71.64%), and ALP (53.18%) in addition to total bilirubin level (50.99%). On the other isle, albumin activity was significantly decreased (*P* < 0.01) by -20.32% relative to the normal control.

The oral supplementation of rutin to DXR-injected animals was associated with a significant drop (*P* < 0.01) in the activities of serum ALT (-35.14%), AST (-38.00%), and ALP (-52.62%) and in the total bilirubin level (-24.95%) without influencing (*P* > 0.05) the serum albumin level (6.79%). Similarly, the oral supplementation of quercetin to DXR-injected rats significantly dropped (*P* < 0.01) the activities of ALT, AST, and ALP recording percent changes of -52.47%, -29.97%, and -71.17%, respectively, while it significantly elevated (*P* < 0.01) the level of albumin (19.10%). The oral supplementation of a combination of rutin and quercetin to DXR-injected rats was associated with a significant drop (*P* < 0.01) in the activities of serum ALT, AST, and ALP by -51.48%, -32.33%, and -62.86%, respectively, and with a significant elevation (*P* < 0.05) in the level of albumin (17.69%). The oral supplementation of a mixture of quercetin and rutin also produced an outstanding decrease in bilirubin level (-18.57%). Quercetin proved to be the most potent in reducing the high ALT and ALP activities by -52.47% and -71.18%, respectively, as well as in increasing the lowered albumin level by 19.10%. Rutin proved to be the most potent in decreasing the high AST activity and bilirubin level by -38.00% and -24.95%, respectively.

### 3.2. Effect on Serum Tumor Marker Level

Data reflecting the influence on serum AFP and CA 19.9 levels by rutin and/or querctin are shown in Table 2. Serum AFP and CA19.9 levels significantly increased (*P* < 0.01) by 154.34% and 126.88%, respectively, in response to the intraperitoneal administration of DXR in Wistar rats. A nonsignificant elevation (*P* > 0.05) in serum AFP by 1.71% and a significant drop (*P* < 0.01) in serum CA19.9 by -26.06% were spotted when the DXR-injected rats were supplemented with rutin. A significant decrease (*P* < 0.05) in AFP level by -21.36% and a highly significant drop (*P* < 0.01) in CA19.9 level by -35.3% were recording after supplementing the DXR-injected rats with quercetin. On other hand, the levels of both AFP and CA19.9 were significantly downregulated (*P* < 0.01) by -46.15% and -53.65%, respectively, upon supplementing the DXR-injected rats with the combination of quercetin and rutin. The general between-group effect on serum levels of AFP and CA19.9 was very significant (*P* < 0.001) as revealed by the one-way ANOVA.

### 3.3. Influence of the Treatments on Liver Antioxidant Defense System and Oxidative Stress

Liver GSH content was significantly downregulated (*P* < 0.01) by -45.90% relative to normal control when DXR was administered intraperitoneally to rats. This effect was reversed by supplementing rutin to DXR-injected rats where a significant upregulation (*P* < 0.01) of GSH content by 66.25% was produced. On the other hand, the supplementation of quercetin alone or together with rutin to the DXR-injected group was associated with a nonsignificant elevation (*P* > 0.05) in the GSH content by 23.01% and 10.06%, respectively.

Liver LPO level was significantly upregulated (*P* < 0.01) upon intraperitoneal administration of DXR to Wistar rats where the recorded percentage change was 60.17% relative to control rats. The supplementation with either rutin or quercetin or their combination caused liver LPO to drop significantly (*P* < 0.05) with quercetin being the most efficient in reducing the elevated LPO by -35.08% (Table 3).

### 3.4. Effect on the Activities of Diverse Antioxidant Enzymes in the Liver of DXR-Injected Rats

Liver GPx activity was highly suppressed (*P* < 0.01) following intraperitoneal administration of DXR to Wistar rats, where the documented percentage change was -31.20%. The oral supplementation of rutin to DXR-injected rats significantly elevated (*P* < 0.01) liver GPx activity by 21.64%. On the other isle, liver GPx activity increased marginally (*P* > 0.05) by 6.98% following oral supplementation of quercetin to DXR-injected rats. A similar marginal increase (*P* > 0.05) in liver GPx activity by 13.48% was observed when rutin and quercetin were co-supplemented to DXR-injected rats (Table 4).

Upon administration of DXR intraperitoneally to Wistar rats, liver GST activity was significantly reduced (*P* < 0.01), where the reported percentage change was -34.50%. The oral supplementation of rutin to DXR-injected rats failed to significantly alter the activity of liver GST (*P* > 0.05) with 15.86% being reported as the percentage change. However, the oral supplementation of quercetin to DXR-injected rats managed to elevate the activity of liver GST in a significant manner (*P* < 0.01) by 43.42%. Further elevation in the percentage change (*P* < 0.01) to 57.50% was observed upon oral cosupplementation of quercetin and rutin (Table 4).

A non-significant impact (*P* > 0.05) was spotted on the activity of liver SOD, with reported percentage change -1.43%, when DXR was intraperitoneally injected to Wistar rats. The oral supplementation of rutin was tied to a significant elevation (*P* < 0.01) in liver SOD activity by 23.90%. Likewise, the activity was significantly upregulated (*P* < 0.01) by 13.88% upon treatment with quercetin. Administering a mixture of quercetin and rutin significantly raised (*P* < 0.01) liver SOD activity by 10.98% (Table 4).

### 3.5. Histopathological Investigations

Normal liver architecture composed of hepatic lobules was presented when normal control rats were given equivalent volumes of vehicles (Figure 1). Each of them has a thin-walled central vein from which the hepatic trabeculae radiate in the direction of the lobule periphery and alternate interchanges with sinusoids around the periphery of each lobule branches of hepatic artery, in addition to hepatic portal vein and bile ductules (Figure 1). Conversely, the liver of DXR-injected rats showed significant changes. Hepatic capsule inflammation and subcapsular hepatocyte cytoplasmic vacuolization (Figures 2(a) and 2(b)), clear cells of hepatocytes (Figure 2(b)), karyomegaly of hepatocytic nuclei (Figure 2(c)), and apoptosis of hepatocytes (Figures 2(c) and 2(d)) are examples of such changes.

When treated with rutin, liver sections of DXR-injected rats manifested the necrosis of sporadic hepatocytes (Figure 3(a)) and fatty change of hepatocytes (Figure 3(b)). Quercetin treatment, on the other hand, resulted in some improvement in the liver histological features if compared to the control rats injected with DXR. Apparently, histopathological changes were lacking (Figures 4(a) and 4(b)) and slight vacuolization of hepatocytes was exhibited (Figure 4(c)). The same outcomes were noticed when the DXR-injected rats were treated with the mixture of quercetin and rutin (Figures 5(a)–5(c)).

The liver histological lesion scores presented in Table 5 depicted that inflammation, necrosis, activated apoptosis, vascularization of hepatocytes, clear cells of hepatocytes, and karyomegaly of hepatocytic nuclei exhibited less scores in quercetin and rutin treated rats than in control rats injected with DXR; the combinatory effect was the most potent. All histological scores exhibited significant effects (*P* < 0.01) when the group injected with DXR was contrasted with the normal control group. With the exception of the effect of rutin on vascularization of hepatocytes, all treated DXR-injected group showed significant improvements of all lesions when compared with the DXR-injected control (Table 6).

### 3.6. Immunohistochemical Investigations

Immunohistochemical staining of p53 showed a weak expression of p53 in the liver of normal rats (Figure 6(a)). On the contrary, the liver of DXR-injected rats exhibited a very high activated expression of p53 illustrated by a dense cytoplasmic brownish color (Figure 6(b)). Conversely, DXR-injected rats treated with rutin (Figure 6(c)) exhibited a weak expression of p53, whereas the DXR-injected rats treated with quercetin showed a weak expression of p53 (Figure 6(d)). Treatment with the mixture of quercetin and rutin demonstrated a moderate expression of p53 in the liver of DXR-injected rats (Figure 6(e)).

Immunohistochemical staining of TNF-*α* demonstrated a weak expression of TNF-*α* in the liver of normal rats (Figure 7(a)). In contrast, a strong activated expression of TNF-*α* (represented by a dense cytoplasmic brownish color) in the liver of DXR-injected rats was demonstrated (Figure 7(b)). However, DXR-injected rats exhibited a weak (Figure 7(c)), moderate (Figure 7(d)), and negative (Figure 7(e)) expression of TNF-*α* when treated with rutin, quercetin, and rutin/quercetin mixture, respectively.

Immunohistochemical staining of Nrf2 demonstrated a mild expression of Nrf2 in the liver of normal rats (Figure 8(a)). Activated expression of Nrf2 was negative in the liver of DXR-injected rats (Figure 8(b)). On the contrary, DXR-injected rats treated with rutin demonstrated strong expression illustrated by dense cytoplasmic brownish color (Figure 8(c)). The liver of DXR-injected rats treated with quercetin demonstrated a mild activated expression of Nrf2 (Figure 8(d)). The liver of DXR-injected rats treated with the mixture presented negative expression of Nrf2 (Figure 8(e)).

Image analysis of immunohistochemical sections indicated a significant increase (*P* < 0.01) of liver p53 expression recording percentage change of 998.41% on injection of DXR. All DXR-injected groups supplemented with rutin or quercetin or their mixture demonstrated a significant drop (*P* < 0.01) in liver p53 reporting percentage changes of -92.47%, -66.37%, and -64.58%, respectively (Table 7).

A significant rise (*P* < 0.01) of liver TNF-*α* expression was induced by the injection of DXR reporting percentage change of 659.36%. All DXR-injected groups supplemented with quercetin and/or rutin exhibited significant drops (*P* < 0.01) in TNF-*α* expression recording percentage changes of -80.70%, -78.59%, and -97.57%, respectively (Table 7).

In contrast to p53 and TNF-*α*, the injection of DXR significantly reduced (*P* < 0.01) liver Nrf2 expression recording percentage of -98.76%. The DXR-injected group supplemented with either rutin or quercetin exhibited a sharp rise (*P* < 0.01) in liver Nrf2 expression recording percentage of 73620% and 14360%, respectively. However, supplementing with both rutin and quercetin failed to elevate liver Nrf2 content in a significant way (*P* > 0.05) although a percentage change of 214% was recorded (Table 7).

## 4. Discussion

While DXR is effective against a range of human malignancies, its toxicity precludes it from being used as a cancer chemotherapeutic agent [18, 56, 57]. Additionally, one of the most serious drawbacks of the anticancer therapy with DXR on the long term is resistance to the chemotherapeutic agent [18].

As demonstrated in this research, DXR enhanced the activities of the cytoplasmic enzyme ALT, the cytoplasmic and mitochondrial enzyme AST, and the membrane-bound enzyme ALP, as well as total bilirubin level. Reduced liver functioning and hepatocellular damage are responsible for these increases. In a DXR-induced hepatotoxicity model, similar high levels of serum indices for hepatocellular damage as well as hepatobiliary deterioration were previously reported [58–61]. The current data are also consistent with those previously published elsewhere [60, 62–65] as elevation of the activities of ALT, AST, and ALP in the serum of rats injected with DXR has been reported. Sathesh et al. [66] also stated that DXR treatment caused tissue damage as well as an increase in enzyme membrane leakage. Thus, our results in accordance with previous publications confirmed that a significant increase of liver cytoplasmic enzymes in the serum takes place as considerable amounts of these enzymes leak to blood stream from necrotic hepatocytes, as a result of DXR-induced toxicity. In addition, the increase in serum ALP activity reflects the damage in bile ductular cells and release of this membrane bound enzyme into blood. The damaging effects of DXR on liver cells may attributed to the stimulation of oxidative stress and inflammation. Both increased levels of LPO and TNF-*α* have important implications of necrosis and damage of liver cells [67–69] (Scheme 2). The current investigation showed that employing rutin and quercetin for the treatment of DXR-injected rats remarkably decreased the raised activities of serum ALT, AST, and ALP and the level of total bilirubin as well. The decrease in these serum biomarkers provides evidence that both rutin and quercetin treatments have profound positive effects on the function and integrity of the liver. In addition, the decrease in ALT, AST, and ALP activities may be secondary to the improvements in liver structural integrity as demonstrated by the results of the histological investigation conducted herein. Oxidative stress, inflammation, and apoptosis suppression by treatments with rutin and quercetin attribute to the amelioration of liver function and structural integrity (Scheme 2).

The present investigation found that DXR-injected animals exhibited elevated levels of serum total bilirubin, which is similar with the results of Liss et al. [70], Ahmed [71], Hozayen et al. [60], Hassan et al. [67], Ahmed et al. [68], and Ahmed et al. [72]. These researchers argued that it is a clear indicator of liver disease and may be caused by bile ductile occlusion induced by portal triad inflammation and fibrosis and/or conjugated bilirubin reflux from necrotic hepatocytes to sinusoids. When DXR-injected rats in the present investigation were treated with rutin or rutin/quercetin mixture, a substantial drop in the elevated serum bilirubin levels resulted; this reflects an improvement in the hepatobiliary system.

According to the current findings, the DXR-injected rats were with significantly reduced levels of serum albumin. Relative to control rats injected with DXR, quercetin and quercetin/rutin-treated rats were with significantly increased albumin level, which is similar to the observations by Hozayen et al. [60] and Ahmed et al. [73]. These investigators documented ameliorative effects of various flavonoids on serum albumin levels in drug- and chemicals-intoxicated rats. The decrease in the concentration of serum albumin herein in DXR-injected rats could be assigned to the impaired synthesis of albumin in the affected hepatic tissue under the oxidative stress and the damaging effects of DXR. The amelioration of serum albumin level, however, could indicate the protecting role of quercetin and quercetin/rutin mixture on the liver maintaining albumin synthesis near normal.

The amelioration of liver function biomarkers in serum resulting from treatment with rutin and quercetin was linked to the enhancement of liver histological architecture and integrity. This synchronization was evidenced by the present results, which indicated less values of histopathological scores including inflammation, necrosis, apoptosis, vacuolization of hepatocytes, clear cells of hepatocytes, and karyomegaly of hepatocytic nuclei when rats injected with DXR were supplemented with rutin and quercetin. With the exception of vascularization of hepatocytes, the effects of rutin and quercetin were quite similar. This can be explained by the elucidation that after the rutin and quercetin administration, sulfates and glucuronides of quercetin were exclusively present in the bloodstream, whereas rutin and quercetin were not detected [74–77]. Because the administration of both rutin and quercetin results in the production of the same metabolites, i.e., sulfates and glucuronides of quercetin, this may attribute the nonsignificant effects between these two treatments.

Returning to our data, DXR-injected rats had higher levels of the tumor indicators CA19.9 and AFP in serum which is in line with the observations by Hozayn et al. [60] but differ from those by Attallah et al. [77] who found that serum AFP and CA 19.9 indicators were nonsignificantly altered by all tested dosages of the hepatotoxin, furfural, in the early identification of hepatocellular carcinoma (HCC).

The elevated level of AFP in serum could have resulted from the greater leakage of newly synthesized AFP from injured hepatocytes into the circulating blood. Additionally, this could be due to increased susceptibility of rats to HCC, as a result of DXR administration [78]. AFP synthesis is restored in moderately differentiated hepatomas in murine regenerative cells, and AFP reexpression occurs in the perinecrotic cell layer in the liver poisoned by various hepatotoxins, according to Abelev [79] and Fahim et al. [78]. Furthermore, increased CA 19.9 levels have been linked to impaired liver function [80]. Nonmalignant conditions such as pancreatitis, cholelithiasis, cholestasis, certain lung disorders, and liver cirrhosis have also been linked to elevated serum CA 19.9 [81]. Additionally, Schlick et al. [82] indicated that the elevated levels of serum CA 19.9 were caused by toxicity associated with Folfirinox treatment of pancreatic cancer. The DXR-treated rats had a marginal increase in serum AFP, which contradicts to the findings of Hozayn et al. [60] who claimed that serum AFP levels were significantly increased after DXR administration alone but were significantly improved when the DXR-injected animals received either rutin or hesperidin.

Supplementing DXR-injected rats with rutin significantly spiked the level of serum CA19.9. The quercetin treatment of DXR-injected rats significantly lowered AFP and CA19.9 values in serum. Baker et al. [83] reported similar findings and indicated that estrogen binding to AFP was prohibited by the flavonols quercetin and kaempferol with an apparent equilibrium dissociation constant of approximately 5 × 10^−7^ M. In a N-nitrosodiethylamine-induced hepatocarcinogenesis model, remodeling of preneoplastic foci was expedited and HCC cells, hyperplastic nodules, in addition to the number of persistent foci were greatly reduced by quercetin treatment [84]. Despite these positive findings, other researchers discovered that in a rat model of heterocyclic amine-induced hepatocarcinogenesis dietary quercetin was able to increase the formation of GST-P-positive foci. Conversely, this investigation focused on GST-P foci rather than on tumor formation as a replacement endpoint [85, 86]. In human HCC cells, quercetin suppresses proliferation and promotes apoptosis in *vitro* [87]. Quercetin was also reported to enhance human HCC cell death induced by radiation [88].

In contrast, supplementing rutin and quercetin to rats injected with DXR significantly reduced both AFP and CA19.9 levels. These results may indicate that rutin and quercetin may have potent effects to improve the levels of these tumor markers and decrease the probability of liver cancer.

The deleterious biochemical and histological changes demonstrated in the DXR-injected rats were linked to a significant rise in the level of liver LPO, as well as to a significant drop in the liver content of GSH and in the activities of antioxidant enzymes (GST, GPx, and SOD).

DXR-induced cellular damage is mediated by the induction of ROS production and attenuation of the antioxidant defense system by DXR as hypothesized by many investigators [60, 89–92]. Those investigators also reported that higher LPO level is linked to liver damage. In the same line, Jagetia and Lalrinengi [93] revealed that DXR's enhanced toxicity in the liver could be attributed to its capacity to deplete GST and to elevate LPO. It was also indicated by the same authors that DXR administration produced time and dose-dependent reduction in the activity of GST. The activity increased when naringin was administered before and after DXR treatment. These results are in consistent with those of Jagetia and Lalnuntluangi [94].

According to Chen et al. [95], rutin at a dose of 1.0 *μ*g/kg bw remarkably inhibit LPO in rat liver and effectively restored GSH content and SOD activity in alcohol-treated rat livers. These results indicate that rutin have a favorable effect in reducing the adverse effect of alcohol and could be used to treat liver injury as a potent antialcoholic agent.

Found in nonedible and edible plants, polyphenolic substances have been shown to have antioxidant activities among other biological effects. Antioxidants, such as flavonoids, behave as reducing agents that act by neutralizing superoxide (O_2_^·-^) and hydroxyl radicals (^·^*OH*) among other oxidizing free radicals. Besides, flavonoids and phenolic compounds have been shown to be powerful suppressors of LPO and thus acting as effective scavengers of peroxyl radicals (ROO^·^). The constituents of orange, including phenols and flavonoids, have the potential to lower oxidative damage by direct and indirect inhibition of free radical excessive production [96].

The preventive effects of rutin and quercetin against liver toxicity were accompanied by a reduction in liver LPO and an increase in GSH concentration, as well as increased GPx, GST, and SOD activities. This is consistent with the findings of Umarani et al. [97], Kebiechc et al. [98], and our previous publications [23, 24]. It is worth mentioning here that apoptosis, *via* an intrinsic pathway, and necrosis, *via* increased membrane lipid peroxidation, are activated by the state of oxidative stress and the excessive liberation of ROS. Thus, employing rutin, quercetin and their combination to relieve the state of oxidative stress and promote the antioxidant defense system may be a key player in suppressing both apoptosis and necrosis (Scheme 2).

The intrinsic pathway leading to apoptosis is essentially mediated by the proapoptotic protein, p53 (Scheme 2). The administration of DXR, in the current study, resulted in high levels of liver p53, which is improved when quercetin or a combination of rutin and quercetin is administered as a treatment. These results are consistent with those of Porteiro et al. [99] and Wang et al. [100] who revealed that antitumor drugs like DXR promote the apoptosis of tumor cells by implementing a mechanism that is mediated through activated p53. Attempting to understand the role of p53 protein in the ability of quercetin to potentiate liver cancer cell apoptosis induced by DXR, Wang et al. examined p53 protein expression in control, quercetin-treated, and quercetin/DXR cotreated cells. The fact that no measurable levels of p53 protein expression were detected in the quercetin-treated cells and that remarkable levels were detected in the quercetin/DXR cotreated cells ruled out the involvement of p53 protein expression. The presented results in this study are also in concurrence with the study of Hassan et al. [67] who found that the two flavonoids naringin and hesperidin have antiapoptotic effects. Accordingly, it can be stated that the antiapoptotic actions of rutin and quercetin may abate the deteriorating effects of DXR on liver function and integrity (Scheme 2).

TNF-*α* (a proinflammatory cytokine) level increased significantly in the serum of rats injected with DXR in the current study. These findings are consistent with those of Shankar et al. [101] and Ahmed et al. [28] who reported augmented levels of cytokine TNF-*α* upon DXR injection, which triggers multiple inflammatory pathways and apoptosis *via* an extrinsic pathway through binding to tumor necrosis factor receptor (TNFR) (Scheme 2). Tangpong et al. [102] demonstrated that TNF-*α* causes mitochondrial dysfunction as a result of its downstream effects, which include increased oxidative stress, TUNEL-positive cell death, cytochrome C release, and caspase 3 activity; all of which have been linked to DXR-induced apoptosis. Nevertheless, cell death induced by TNF-*α* is mainly apoptotic although necrosis may also take part [67, 103] (Scheme 2). When DXR-injected rats were treated with rutin and quercetin in the present study, the elevated TNF-*α* expression in the liver dropped significantly. Thus, it can be suggested that the anti-inflammatory, antiapoptotic and antinecrotic effects of rutin and quercetin in DXR-injected rats may be attributed at least in part to the suppressing effects on TNF-*α*.

Nrf2 is an emerging regulator of cellular resistance to ROS (Scheme 2). It activates the basal as well as induced expressions of antioxidant response element- (ARE-) dependent genes to control the physiological and pathophysiological outcomes of oxidant exposure [104]. In the present study, liver Nrf2 expression was significantly decreased in the DXR-injected group as compared to the normal control and was significantly increased following administration of rutin and quercetin in rats injected with DXR-injected rats. There is accumulating evidence from previous publications that the expression of antioxidant ARE genes, which also exert anti-inflammatory actions, is regulated mainly by the transcription factor Nrf2 [105] (Scheme 2). Thus, the increase in liver Nrf2 expression may be a key player in mediating the antioxidant and anti-inflammatory effects exerted by rutin and quercetin in Wistar rats with DXR-induced hepatotoxicity (Scheme 2).

## 5. Conclusions

In conclusion, quercetin and/or rutin was proved to provide potential chemopreventive effects against hepatotoxicity induced by DXR through suppressing oxidative stress, inflammation, and apoptosis, as well as through modulating effects of Nrf2.

## Figures and Tables

**Scheme 1:** Schematic diagram of animal groups and employed experimental design.

**Figure 1:** Photomicrograph of liver section in an untreated rat indicating normal liver architecture composed of a central vein (CV) with thin walls and normal hepatocytes with narrow intercellular sinusoids (S) (H&E; ×400).

**Figure 2:** Photomicrographs of liver sections in rats injected with DXR indicating inflammation (IF) of hepatic capsule (a), cytoplasmic vacuolization (V) of subcapsular hepatocytes (a, b), clear cells of hepatocytes (CC) (b), apoptosis (AP) of hepatocytes (c, d), and karyomegally (K) of hepatocytic nuclei (c) (H&E; ×400).

**Figure 3:** Photomicrographs of liver sections in rats injected with DXR after supplementing with rutin indicating necrosis (NC) of spaoradic hepatocytes (a) and fatty change (F) of hepatocytes (b) (H&E; ×400).

**Figure 4:** Photomicrographs of liver sections in rats injected with DXR after supplementing with quercetin indicating nearly normal structure of liver tissue with no histological changes (a, b) and slight vacuolization (V) of hepatocytes (c) (H&E; ×400).

**Figure 5:** Photomicrographs of liver sections in rats injected with DXR after supplementing with a combination of quercetin and rutin indicating slight vacuolization (V) of hepatocytes (a) and almost normal structure of the liver tissue with no histological changes (b, c) (H&E; ×400).

**Figure 6:** Photomicrographs of immunohistochemical sections of liver for detection of p53 showing weak expression in normal rats (a), very strong staining expression (immunopositivity indicated by brownish color) in DXR administered rats (b), weak expression in DXR administered rats treated with rutin (c), and moderate expression in DXR administered rats treated with quercetin (d) and its combination with rutin (6e) (×100).

**Figure 7:** Photomicrographs of immunohistochemical sections of liver for detection of TNF-*α* showing weak expression of in normal rats (a), strong expression (immunopositivity indicated by brownish color) in DXR-injected rats (b), weak expression in DXR-injected rats treated with rutin (c) and quercetin (d), and negative expression in DXR-injected rats treated with mixture of rutin and quercetin (e) (×100).

**Figure 8:** Photomicrographs of immunohistochemical sections of liver for detection of Nrf2 showing weak expression of Nrf2 in normal rats (a), very weak expression in DXR-injected rats (b), strong expression (immunopositivity indicated by brownish color) in DXR-injected rats treated with rutin (c), mild expression (immunopositivity indicated by brownish color) in DXR-injected rats treated with quercetin (d), and very weak expression in DXR-injected rats treated with a mixture of rutin and quercetin (e) (×100).

**Scheme 2:** Schematic figure showing the mechanisms of action of rutin and quercetin to counter DXR hepatotoxicity via oxidative stress, inflammation and apoptosis suppression and antioxidant defense mechanism promotion through the Nrf2 signaling pathway. DXR: doxorubicin; Keap1: Kelch-like ECH-associated protein 1; ARE: antioxidant response element; Nrf2: nuclear factor E2-related factor 2; ROS: reactive oxygen species; TNFR: tumor necrosis factor-*α* receptor.

**Table 1:** Serum parameters related to liver function in normal rats and in rats injected with DXR (without and with the supplementation of rutin and/or quercetin).

Parameter					
Groups	ALT (U/L)	AST (U/L)	ALP (U/L)	Bilirubin (mg/dL)	Albumin (g/dL)
Normal control	57.50 ± 4.06	152.25 ± 5.68	180.50 ± 0.12	0.35 ± 6.40	3.12 ± 0.04
DXR-injected control group	101.00 ± 16.69^++^	261.33 ± 18.18^++^	276.50 ± 19.23^++^	0.53 ± 5.16^++^	2.48 ± 0.18^++^
DXR-injected group supplemented with rutin	65.50 ± 4.52^∗∗^	162.00 ± 1.80^∗∗^	131.00 ± 5.39^∗∗^^$^	0.40 ± 4.93^∗∗^	2.65 ± 0.14
DXR-injected group supplemented with quercetin	48.00 ± 4.28^∗∗^	183.00 ± 9.12^∗∗^	79.66 ± 2.44^∗∗^	0.56 ± 2.84^$$^	2.96 ± 0.09^∗∗^
DXR-injected group supplemented with rutin and quercetin	49.00 ± 4.75^∗∗^	176.83 ± 15.61^∗∗^	102.66 ± 7.18^∗∗^	0.43 ± 0.10^∗^	2.92 ± 0.02^∗^
*F*-probability	*P* < 0.001	*P* < 0.001	*P* < 0.001	*P* < 0.001	*P* < 0.001

Values are *M* ± SE (*n* = 6). ^+^*P* < 0.05, ^++^*P* < 0.01: the DXR-injected control group versus (vs.) normal control. ^∗^*P* < 0.05, ^∗∗^*P* < 0.01: the DXR-injected groups treated with rutin and/or quercetin vs. DXR-injected control group. ^$^*P* < 0.05, ^$$^*P* < 0.01: the DXR-injected groups treated with rutin or quercetin alone vs. DXR-injected group treated with rutin and quercetin mixture.

**Table 2:** Serum AFP and CA19.9 levels in normal rats and in rats injected with DXR (without and with the supplementation of rutin and/or quercetin).

Parameter		
Group	AFP (ng/mL)	CA19.9 (U/L)
Normal control	0.46 ± 0.04	119.17 ± 2.36
DXR-injected control group	1.17 ± 0.03^++^	270.37 ± 36.93^++^
DXR-injected group supplemented with rutin	1.19 ± 0.05^$$^	199.9 ± 0.72^∗∗^^$$^
DXR-injected group supplemented with quercetin	0.92 ± 0.16^∗^^$^	174.8 ± 4.92^∗∗^^$^
DXR-injected group supplemented with rutin and quercetin	0.63 ± 0.05^∗∗^	125.3 ± 1.74^∗∗^
*F*-probability	*P* < 0.001	*P* < 0.001

Values are *M* ± SE (*n* = 6). ^+^*P* < 0.05, ^++^*P* < 0.01: the DXR-injected control group vs. normal control. ^∗^*P* < 0.05, ^∗∗^*P* < 0.01: the DXR-injected groups treated with rutin and/or quercetin vs. DXR-injected control group. ^$^*P* < 0.05, ^$$^*P* < 0.01: the DXR-injected groups treated with rutin or quercetin alone vs. DXR-injected group treated with rutin and quercetin mixture.

**Table 3:** Liver GSH content and LPO in normal rats and in rats injected with DXR (without and with the supplementation of rutin and/or quercetin).

Parameter		
Group	GSH (nmole/100 mg tissue)	LPO (nmole MDA/100 mg tissue/hr)
Normal control	118.91 ± 5.11	17.55 ± 1.05
DXR-injected control group	64.32 ± 6.54^++^	28.11 ± 0.87^++^
DXR-injected group supplemented with rutin	106.95 ± 14.40^∗∗^^$$^	20.41 ± 1.57^∗∗^
DXR-injected group supplemented with quercetin	79.13 ± 8.04	18.25 ± 1.40^∗∗^
DXR-injected group supplemented with rutin and quercetin	70.80 ± 4.65	20.35 ± 0.87^∗∗^
*F*-probability	*P* < 0.001	*P* < 0.001

Values are *M* ± SE (*n* = 6). ^+^*P* < 0.05, ^++^*P* < 0.01: the DXR-injected control group vs. normal control. ^∗^*P* < 0.05, ^∗∗^*P* < 0.01: the DXR-injected groups treated with rutin and/or quercetin vs. DXR-injected control group. ^$^*P* < 0.05, ^$$^*P* < 0.01: the DXR-injected groups treated with rutin or quercetin alone vs. DXR-injected group treated with rutin and quercetin mixture.

**Table 4:** GPx, GST, and SOD activities in the liver of normal rats and rats injected with DXR (without and with the supplementation of rutin and/or quercetin).

Parameter			
Groups	GPx (mU/100 mg tissue)	GST (mU/100 mg tissue)	SOD (mU/100 mg tissue)
Normal control	101.91 ± 8.61	105.40 ± 4.72	112.91 ± 1.68
DXR-injected control group	70.10 ± 2.32^++^	69.03 ± 4.63^++^	111.29 ± 1.35
DXR-injected group supplemented with rutin	85.28 ± 5.29^∗^	79.98 ± 5.24^$^	137.89 ± 2.63^∗∗^^$$^
DXR-injected group supplemented with quercetin	75.60 ± 5.30	99.10 ± 14.26^∗^	126.74 ± 4.77^∗∗^
DXR-injected group supplemented with rutin and quercetin	79.56 ± 1.51	108.72 ± 6.64^∗^	123.51 ± 3.35^∗∗^
*F*-probability	*P* < 0.001	*P* < 0.01	*P* < 0.001

Values are *M* ± SE (*n* = 6). ^+^*P* < 0.05, ^++^*P* < 0.01: the DXR-injected control group vs. normal control. ^∗^*P* < 0.05, ^∗∗^*P* < 0.01: the DXR-injected groups treated with rutin and/or quercetin vs. DXR-injected control group. ^$^*P* < 0.05, ^$$^*P* < 0.01: the DXR-injected groups treated with rutin or quercetin alone vs. DXR-injected group treated with rutin and quercetin mixture.

**Table 5:** Histological lesion scores of liver in normal rats and in rats injected with DXR (without and with the supplementation of rutin and/or quercetin).

Histopathological changes	Score	Normal control	DXR-injected control	DXR-injected group treated with rutin	DXR-injected group treated with quercetin	DXR-injected group treated with rutin and quercetin
Inflammation	0	6 (100.00%)	2 (33.33%)	4 (66.66%)	5 (83.33%)	6 (100.00%)
	I	—	2 (33.33%)	2 (33.33%)	1 (16.66%)	—
	II	—	2 (33.33%)	—	—	—
	III	—	—	—	—	—
Necrosis	0	6 (100.00%)	—	4 (66.66)	6 (100.00%)	6 (100.00%)
	I	—	3 (50.00%)	2 (33.33%)	—	—
	II	—	1 (16.66%)	—	—	—
	III	—	2 (33.33%)	—	—	—
Activated apoptosis	0	6 (100.00%)	2 (33.33%)	5 (83.33%)	6 (100.00%)	6 (100.00%)
	I	—	2 (33.33%)	1 (16.66%)	—	—
	II	—	2 (33.33%)	—	—	—
	III	—	—	—	—	—
Vacuolization of hepaocytes	0	6 (100.00%)	—	2 (33.33%)	4 (66.66)	5 (83.33%)
	I	—	1 (16.7%)	—	1 (16.66%)	—
	II	—	1 (16.7%)	2 (33.33%)	—	1 (16.66%)
	III	—	4 (66.66)	2 (33.33%)	1 (16.66%)	—
Clear cells of hepatocytes	0	6 (100.00%)	2 (33.33%)	6 (100.00%)	6 (100.00%)	6 (100.00%)
	I	—	2 (33.33%)	—	—	—
	II	—	2 (33.33%)	—	—	—
	III	—	—	—	—	—
Karyomegaly of hepatocytic nuclei	0	6 (100.00%)	2 (33.33%)	5 (83.33%)	6 (100.00%)	6 (100.00%)
	I	—	1 (16.66%)	1 (16.66%)	—	—
	II	—	1 (16.66%)	—	—	—
	III	—	2 (33.33%)	—	—	—

Number of animals in each group is 6. 0: means absence of lesion; I: means mild; II: means moderate; and III: means severe. The % in brackets is the percentage of animals in every assigned grade.

**Table 6:** Effect on histological lesion scores of liver in normal rats and in rats injected with DXR (without and with the supplementation of rutin and/or quercetin).

Lesion score						
Groups	Inflammation	Necrosis	Activated apoptosis	Vascularization of hepatocytes	Clear cells of hepatocytes	Karyomegaly of hepatocytic nuclei
Normal control	0.000 ± 0.000	0.000 ± 0.000	0.000 ± 0.000	0.000 ± 0.000	0.000 ± 0.000	0.000 ± 0.000
DXR-injected control group	1.000 ± 0.365^++^	1.333 ± 0421^++^	1.000 ± 0.365^++^	2.500 ± 0.341^++^	1.000 ± 0.365^++^	1.500 ± 0.562^++^
DXR-injected group supplemented with rutin	0.333 ± 0.210^∗^	0.333 ± 0.210^∗∗^	0.161 ± 0.166^∗∗^	1.666 ± 0.557^$^	0.000 ± 0.000^∗∗^	0.166 ± 0167^∗∗^
DXR-injected group supplemented with quercetin	0.000 ± 0.000^∗∗^	0.000 ± 0.000^∗∗^	0.000 ± 0.000^∗∗^	0.666 ± 0.494^∗∗^	0.000 ± 0.000^∗∗^	0.000 ± 0.000^∗∗^
DXR-injected group supplemented with rutin and quercetin	0.000 ± 0.000^∗∗^	0.000 ± 0.000^∗∗^	0.000 ± 0.000^∗∗^	0.333 ± 0.333^∗∗^	0.000 ± 0.000^∗∗^	0.000 ± 0.000^∗∗^
*F*-probability	*P* < 0.01	*P* < 0.001	*P* < 0.01	*P* < 0.001	*P* < 0.001	*P* < 0.01

Values are *M* ± SE (*n* = 6). ^+^*P* < 0.05, ^++^*P* < 0.01: the DXR-injected control group vs. normal control. ^∗^*P* < 0.05, ^∗∗^*P* < 0.01: the DXR-injected groups treated with rutin and/or quercetin vs. DXR-injected control group. ^$^*P* < 0.05: the DXR-injected groups treated with rutin or quercetin alone vs. DXR-injected group treated with rutin and quercetin mixture.

**Table 7:** Liver p53, TNF-*α*, and Nrf2 in normal rats and in rats injected with DXR (without and with the supplementation of rutin and/or quercetin).

Parameter			
Group	p53 (% area)	TNF-*α* (% area)	Nrf2 (% area)
Normal control	7.56 ± 0.74	3.74 ± 0.83	4.02 ± 0.002
DXR-injected control group	83.04 ± 5.61^++^	28.40 ± 5.93^++^	0.05 ± 0.0002^++^
DXR-injected group supplemented with rutin	6.25 ± 1.06^∗∗^^$$^	5.48 ± 0.68^∗∗^	36.86 ± 1.67^∗∗^^$$^
DXR-injected group supplemented with quercetin	27.93 ± 3.89^∗∗^	6.08 ± 0.08^∗∗^	7.23 ± 0.001^∗∗^^$$^
DXR-injected group treated with rutin and quercetin	29.41 ± 4.38^∗∗^	0.69 ± 0.15^∗∗^	0.157 ± 0.001
*F* probability	*P* < 0.001	*P* < 0.001	*P* < 0.001

Values are *M* ± SE (*n* = 6). ^+^*P* < 0.05, ^++^*P* < 0.01: the DXR-injected control group vs. normal control. ^∗^*P* < 0.05, ^∗∗^*P* < 0.01: the DXR-injected groups treated with rutin and/or quercetin vs. DXR-injected control group. ^$^*P* < 0.05, ^$$^*P* < 0.01: the DXR-injected groups treated with rutin or quercetin alone vs. DXR-injected group treated with rutin and quercetin mixture.

## Data Availability

All data are available from the corresponding author under reasonable request.

## Abbreviations

AFP: Alpha fetoprotein
ALP: Alkaline phosphatase
ALT: Alanine transaminase
ANOVA: Analysis of variance
AST: Aspartate transaminase
ARE: Antioxidant response element
CA19.9: Carbohydrate antigen 19.9
CMC: Carboxymethyl cellulose
DNA: Deoxyribonucleic acid
DXR: Doxorubicin
ELISA: Enzyme-linked immunosorbent assay
Fe^+2^: Ferrous iron
GPx: Glutathione peroxidase
GSH: Glutathione
GST: Gluathione-S-transferase
H&E: Hematoxylin and eosin
Keap1: Kelch-like ECH-associated protein 1
kg bw: Kilogram body weight
LPO: Lipid peroxidation
LSD: Least significant difference
*M* ± SEM: Mean ± standard error of mean
MDA: Malondialdehyde
min: Minutes
NCI: National Cancer Institute
Nrf2: Nuclear factor erythroid 2–related factor 2
p53: Apoptotic protein 53
PBS: Phosphate buffer saline
PCD: Programmed cell death
RNS: Reactive nitrogen species
ROS: Reactive oxygen species
rpm: Round per min
SOD: Superoxide dismutase
TNF-*α*: Tumor necrosis factor-*α*
TNFR: Tumor necrosis factor-*α* receptor
UV: Ultraviolet radiation
vs: Versus.
